The article "A Computer-Aided Diagnosis System Using Deep Learning for Multiclass Skin Lesion Classification" was published in 2021. Journal: Comput Intell Neurosci.

# A Computer-Aided Diagnosis System Using Deep Learning for Multiclass Skin Lesion Classification

**DOI:** 10.1155/2021/9619079

**Published:** 2021-12-06

**Authors:** Mehak Arshad, Muhammad Attique Khan, Usman Tariq, Ammar Armghan, Fayadh Alenezi, Muhammad Younus Javed, Shabnam Mohamed Aslam, Seifedine Kadry

**Affiliations:** ^1^Department of Computer Science, HITEC University Taxila, Taxila, Pakistan; ^2^College of Computer Engineering and Science, Prince Sattam Bin Abdulaziz University, Al-Kharaj, Saudi Arabia; ^3^Department of Electrical Engineering, Jouf University, Sakaka 75471, Saudi Arabia; ^4^Department of Information Technology, College of Computer and Information Sciences, Majmaah University, Al-Majmaah 11952, Saudi Arabia; ^5^Faculty of Applied Computing and Technology, Noroff University College, Kristiansand, Norway

## Abstract

In the USA, each year, almost 5.4 million people are diagnosed with skin cancer. Melanoma is one of the most dangerous types of skin cancer, and its survival rate is 5%. The development of skin cancer has risen over the last couple of years. Early identification of skin cancer can help reduce the human mortality rate. Dermoscopy is a technology used for the acquisition of skin images. However, the manual inspection process consumes more time and required much cost. The recent development in the area of deep learning showed significant performance for classification tasks. In this research work, a new automated framework is proposed for multiclass skin lesion classification. The proposed framework consists of a series of steps. In the first step, augmentation is performed. For the augmentation process, three operations are performed: rotate 90, right-left flip, and up and down flip. In the second step, deep models are fine-tuned. Two models are opted, such as ResNet-50 and ResNet-101, and updated their layers. In the third step, transfer learning is applied to train both fine-tuned deep models on augmented datasets. In the succeeding stage, features are extracted and performed fusion using a modified serial-based approach. Finally, the fused vector is further enhanced by selecting the best features using the skewness-controlled SVR approach. The final selected features are classified using several machine learning algorithms and selected based on the accuracy value. In the experimental process, the augmented HAM10000 dataset is used and achieved an accuracy of 91.7%. Moreover, the performance of the augmented dataset is better as compared to the original imbalanced dataset. In addition, the proposed method is compared with some recent studies and shows improved performance.

## 1. Introduction

The development of skin cancer has risen throughout the previous decade [1]. Ultraviolet rays in the sun damage the skin over time and cause cancer cells to develop [2]. Usually, such conditions have hidden risks that lead to a lack of confidence and psychological distress in humans and to skin cancer risks. Several types of skin cancer exist, including basal cells, melanoma, actinic keratosis, and squamous cell carcinoma [3]. The squamous cell carcinoma is contrasted against actinic keratosis (solar keratosis) [4]. Each year, the incidence rate of both melanoma and nonmelanoma continues to grow [2]. The deadliest form of skin cancer is melanoma and quickly spread to other body parts due to the malignancy of neural crest neoplasia of melanocytes [5].

In the United States, almost 5.4 million new cases of skin cancer are detected each year. Due to melanoma, more than 10,000 deaths are registered every year in the USA [6]. In the USA, 104,350 new cases of skin cancers were diagnosed during the year 2019, where the numbers of deaths were 7230. In the year 2020, 196,060 Americans are diagnosed with melanoma. According to these facts, melanoma cases are increasing approximately 2% [7]. Recently, in the year 2021, 207.39 K peoples are diagnosed with skin cancer whereas the numbers of deaths are 70.18 K. According to the facts, when the lesion is detected earlier, the survival rate increases approximately 98% [7]. The summary of diagnoses and deaths due to skin cancer is illustrated in Figure 1.

Dermatologists diagnose malignant lesions via a dermoscopic visual examination technique [8]. Diagnosis of skin cancer using dermoscopy is challenging due to various textures and wounds [9]. However, the manual inspection of dermoscopic images makes it difficult to diagnose skin cancer with better accuracy. The accuracy of the lesion diagnosis depends on the dermatologist's experience [9]. Few other techniques are available for diagnosing skin cancer, such as biopsy [7] and macroscopic [10]. Due to the complex nature of skin lesions, the clinical methods need more attention and time [11, 12].

The computer-based detection (CAD) techniques are introduced by several researchers in medical imaging [7, 13]. They introduced CAD techniques for several cancers such as skin cancer [14], brain tumor [15, 16], lung cancer [17, 18], COVID-19 [19, 20], and more [21–23]. A simple CAD technique consists of four key steps such as preprocessing of input images, detection of infected parts, features extraction, and classification. A computerized method can be helpful as a second opinion for dermatologists to verify the manual diagnosis results [8]. The advancement in machine learning, like deep learning, has shown much achievement in medical imaging in the last couple of years. Convolutional Neural Network (CNN) is a form of deep learning used for automated features extraction [6]. A convolutional neural network is a computer vision technique that automatically distinguishes and recognizes images' features [24]. Due to its high accuracy, it has attracted interest in medical image processing, agriculture, biometric, and surveillance, to name a few. A simple CNN typically entails a series of layers such as a convolutional layer, ReLU layer [25], normalization layer, pooling layer [26], fully connected layer, and Softmax layer [27]. In many techniques, researchers used some pretrained deep learning models for the classification tasks. A few publically available pretrained deep learning models are AlexNet, VGG, GoogleNet, InceptionV3, and ResNet to name a few [28]. They used these models through transfer learning [7]. Few researchers used feature selection and fusion techniques to improve recognition accuracy [29, 30].

The computer-aided diagnostic systems can allow dermatologists and physicians to make decisions, decrease diagnostic costs, and increase diagnostics reliability [31]. An automated skin lesion identification mechanism is challenging due to several challenges such as changing appearance and imbalanced datasets to name a few [32]. Chaturvedi et al. [6] presented an automated framework for multiclass skin cancer classification. Five steps were involved in the presented method: dataset preprocessing, classification models (pretrained deep learning), fine-tuning, feature extraction, and performance evaluation. During the evaluation process, it is noted that the maximum accuracy of 93.20% was achieved for an individual model (ResNet-101), whereas a complete precision of 92.83% was performed on the ensemble model (InceptionResNetV2 + ResNet-101). In the end, they concluded that the training of deep learning models with the best setup of hyperparameters could be performed better than even ensemble models. Hsin et al. [33] presented the automatic lightweight diagnostic algorithm for skin lesion diagnosis. The presented algorithm was more reliable, feasible, and easy to use. For the experimental process, the HAM10000 dataset was used and achieved an accuracy of 85.8%. Besides, this method was tested on a five-class KCGMH dataset and achieved an accuracy of 89.5%. Kumar et al. [9] presented an automated electronic device. They considered numerous challenges such as skin cancer injuries, skin colors, asymmetric skin, and the shape of the area affected. They used fuzzy C-means to divide homogeneous image regions. Then, some texture features are extracted and trained with the Differential Evolution (DE) algorithm. The experimental process was conducted on HAM10000 and achieved an accuracy of 97.4%.

Afshar et al. [8] presented a computerized method for lesion localization and identification. For the lesion localization, they used RCNN architecture and extract deep features. Later, the best features are selected using Newton-Raphson (IcNR) and artificial bee colony (ABC) optimization. Daghrir et al. [5] developed a hybrid approach for diagnosing suspect lesions that may be checked for melanoma skin cancer. They used a coevolutionary neural network and two classical classifiers in three different methods. Shayini [2] presented a classification framework using geometric and textural information. They used ANN for the final features classification. Results showed improved accuracy as compared to the existing techniques. Akram et al. [7] presented deep learning-based lesion segmentation and classification process. They used Mask RCNN architecture for lesion segmentation. Later, a 24-layered CNN architecture was designed for the multiclass skin lesion classification.

Moreover, many other techniques are introduced such as deep learning and improved moth-flame optimization [34], teledermatology-based architecture [35], hierarchical three-step deep framework [35], and more [36, 37].

### 1.1. Challenges

Several challenges affect the multiclass lesion classification accuracy. As compared to binary class classification, the multiclass problem is a complex and challenging recognition process. The following challenges are considered in this research work:

- Classifying multiple skin lesions into a correct class is challenging due to the high similarity among different lesions.
- The imbalanced dataset classes increase the probability of a higher sample class.
- Multiclass skin lesion types have similar shapes, colors, and textures, which also extract similar features. In the later stage, those features are classified into an incorrect skin class.
- In the fusion step, multiproperties features are fused in one matrix for better accuracy, but it is a high chance that several redundant features are also added. This kind of problem later increases the computational time.
- In the feature extraction step, several essential features are also removed, which may cause a problem of misclassification. Therefore, a good feature optimization technique is required [38].

### 1.2. Major Contributions

In this work, an automated technique has been proposed for multiclass skin lesion classification. The significant contributions in this work are as follows:

- Intraclass pixel change operations are implemented for data augmentation based on the left to right flip, up-to-down flip, and rotation at 90 degrees. This step shifts entire image pixels for differentiating the images from each other for a fair training of a deep model.
- A modified serial-based approach is proposed for the fusion of extracted deep features.
- A novel skewness-controlled SVR approach is proposed for the best feature selection. The best-selected features are finally classified using supervised learning algorithms.

The rest of the manuscript is organized in the following order.  Section 2 presented the proposed methodology including deep feature, selection of best features, and fusion process. Results and comparisons with existing techniques are presented in Section 3. Finally, the manuscript is concluded in Section 4.

## 2. Proposed Methodology

For the multiclass skin lesion classification, a new framework was proposed using deep learning and features selection. The proposed framework consists of a series of steps such as data augmentation, model fine-tuning, transfer learning, feature extraction, the fusion of extracted features, and selection of best features. In the augmentation phase, three operations are performed: rotate 90, right-left flip, and up and down flip. In the fine-tuning model step, two models are opted, such as ResNet-50 and ResNet-101, and updated their layers. Later, transfer learning is applied to train both fine-tuned deep models on augmented datasets. In the subsequent step, features are extracted and performed fusion using a modified serial-based approach. Finally, the fused vector is further enhanced by selecting the best features using the skewness-controlled SVR approach. The main architecture diagram of the proposed framework is illustrated in Figure 2.

### 2.1. Data Augmentation

Data augmentation is a vital information extension approach in machine learning (ML). Data augmentation showed much importance in deep learning due to a massive amount of data for training a model. In this article, the HAM10000 dataset is selected for the experimental process. This dataset consists of seven highly imbalanced classes. Initially, the HAM10000 dataset includes more than 10,000 images of seven skin classes such as 6705 images of melanocytic nevi, 1113 images in melanomas, 1099 images in benign keratoses, 514 images in basal cell carcinomas, 327 images of actinic keratoses, 142 images in vascular lesions, and 115 images in dermatofibromas [39]. From this information, it is noted that few classes are highly imbalanced; therefore, it is essential to balance this dataset. On imbalanced datasets, the deep learning models are not trained for better performance. A few sample images are shown in Figure 3.

Three operations are performed in the data augmentation phase: rotate 90, right-left flip (LR), and up and down flip (UD). These operations are applied multiple times until the number of images in each class reached 6000. In the end, the numbers of images in the newly updated dataset are 42,000, which are previously 10,000. Mathematically, these operations are performed as follows.

Consider an image dataset *ρ*={*a*_1_,…, *a*_*k*_}  [40], where *a*_*k*_ ∈ *U*  is an example image from the dataset. Let *a*_*k*_ have fully *N* pixels; then, the homogeneous pixel matrix coordinates ∁_*k*_ or *a*_*k*_ is defined as follows:

(1) $$\begin{array}{c} {∁}_{K}=\left[\begin{array}{ccc} Y_{1} & Z_{1} & 1\\ Y_{2} & Z_{2} & 1\\ \vdots & \vdots & 1\\ Y_{n} & Z_{n} & 1 \end{array}\right], \end{array}$$

where each row of single-pixel indicates the exact coordinates. Consider that the size of an input image is 256 × 256 × 3, represented by *U*_*i*,*j*,*k*_ having *ith* rows, *j* th columns, and *k* th channels, where *U*_*i*,*j*_ ∈ *R*^*i*×*j*^. The flip-up (UD) operation is formulated as follows [41]:

(2) $$\begin{array}{c} U^{t}=\;U_{j,i}, \end{array}$$

where *U*^*t*^ denotes the transposition of the original image. This image is further updated as follows:

(3) $$\begin{array}{c} U^{V}=\;U_{\left(m+1-i\right)j}, \end{array}$$

where *U*^*V*^ denotes the vertical flip image. The horizontal flip (LR) operation is performed as follows:

(4) $$\begin{array}{c} U^{H}=\;U_{i\left(n+1-j\right)}, \end{array}$$

where *U*^*H*^ denotes the horizontal flip image. The third operation, named rotate 90, is formulated as follows:

(5) $$\begin{array}{c} \text{Rot}=\left[\begin{array}{ccc} \cos\;\beta & -\sin\;\beta & 0\\ \sin\;\beta & \cos\;\beta & 1\\ 0 & 0 & 1 \end{array}\right], \end{array}$$

where Rot denotes the rotation matrix of the image. Visually, these operations are illustrated in Figure 4. This figure shows that three operations are performed on each original image: vertical flip (UD), horizontal flip (LR), and rotate 90.

### 2.2. Convolutional Neural Networks

A convolutional neural network (CNN) is a computer vision technique that automatically distinguishes and recognizes images' features [24]. A simple CNN architecture for image classification is illustrated in Figure 5. In this figure, skin lesion images are considered as input, passed to the convolutional layer. In this layer, weights are transformed into features that are further refined into the pooling layer. Later, the features are transformed into 1D in a fully connected layer. The features of this layer are finally classified through the Softmax layer.

### 2.3. Transfer Learning

Transfer learning is a technique to define applied knowledge based on one or more source activities. Consider a domain *M* consisting of two parts:

(6) $$\begin{array}{c} M=\left\{z,\;Q\left(Z\right)\right\}, \end{array}$$

where *y* is a feature space, and the distribution is marginal:

(7) $$\begin{array}{c} q\left(Z\right),\;Z=\;\left\{z_{1},\ldots .,z_{n}\right\},z_{i}\in Z. \end{array}$$

Given a two-component task *U* and *X*,

(8) $$\begin{array}{c} U=\;\left\{\varphi ,\;Q\left(X|Z\right)\right\}=\left\{\varphi ,\delta \right\};\;\\ X=\;\left\{x_{1},\ldots ,x_{n}\right\},\;\;x_{i}\in \varphi , \end{array}$$

where *φ* is label space containing a prediction function; then, *δ* is trained as

(9) $$\begin{array}{c} \left(x_{i},z_{i}\right),\;z_{i}\in Z,x_{i}\in \varphi . \end{array}$$

Each vector of features in the *M* domain and *δ* represents an appropriate label.

(10) $$\begin{array}{c} \delta \left(x_{i}\right)=\left(z_{i}\right). \end{array}$$

Suppose the source domain *M*_*S*_ and an objective domain *M*_*T*_, where *M*={*z*,  *Q*(*Z*)} and the task is *U*_*S*_ and *U*_*T*_, where *U*= {*φ*, *Q*(*φ|Z*)}. Hence, TL is defined as follows:

- *y*_*S*_ ≠ *y*_*T*_: different feature space
- *Q*(*Z*_*s*_) ≠ *Q*(*Z*_*T*_): different marginal possibilities
- *φ*_*S*_ ≠  *φ*_*T*_: different label spaces
- *Q*(*Z*_*S*_*|Y*_*S*_) ≠ *Q*(*Z*_*T*_*|Y*_*T*_): different conditional probabilities

Visually, this process is illustrated in Figure 6. This figure describes that the ImageNet dataset used as source data has 1000 object classes. After transferring knowledge of the source model to the target model, the weights and labels are updated according to the target dataset. The HAM10000 skin cancer dataset is utilized as a target dataset with seven skin classes in this work.

### 2.4. Fine-Tuned ResNet-50 Deep Features

Residual Network (ResNet) is a traditional neural network model for many computer vision tasks utilized as an integrated network element. The network has a depth of 50 layers and a size of 224 × 224  pixels in the input [42]. When it comes to residual learning functions, ResNet may reformulate network layers given an input mapping reference. The layers are stacked directly within ResNet. The basic idea of ResNet-50 is to use identity mapping to anticipate what is required to obtain the final prediction of previous layer output [43]. ResNet-50 reduces the disappearing gradient effect by applying an alternative bypass shortcut. It may help the model overcome the overfitting training problem. Visually, it is shown in Figure 7.

Moreover, a complete architecture is also given in Figure 8. This figure describes that five residual blocks are used in this network, and in each residual block, multiple layers are added to convolve hidden layer features. Overall, this network includes 50 deep layers with a 7 × 7  input layer receptive field, followed by a max-pooling layer of 3 × 3 kernel size.

The last fully connected (FC) layer is removed, and a new FC layer is added in the fine-tuning process. Then, the new FC layer is connected with the Softmax layer and final classification output layer. The fine-tuned architecture is shown in Figure 9. This figure describes that the augmented skin lesion dataset is considered an input to this network, and in the output, seven classes of different skin cancer types are gotten. After this, the TL technique is employed to train this network, and a new modified network is obtained. In the training process, the following parameters are initialized; for example, the learning rate is 0.0001, the epochs are 100, the minibatch size is 64, and the learning method is Stochastic Gradient Descent (SGD). Features are extracted from the global average pooling layer, which is later utilized for the classification process. The dimension of an extracted feature on this layer is *N* × 2048, where *N* denotes the dermoscopy images.

### 2.5. Fine-Tuned ResNet-101 Deep Features

ResNet-101 consists of 104 layers composed of 33 squares, of which the previous blocks use 29 squares directly [44].  Figure 10 shows a brief description of the ResNet-101 CNN model. In this figure, it is described that the output of the first residual block is 112 × 112. After the first convolutional layer, a max-pooling layer is added of filter size 3 × 3 and stride 2. Using the same sequence, four more residual blocks are added, and each block consists of several layers, as given in Figure 11. This model was initially trained on the ImageNet dataset; therefore, the output was 1000D.

In this work, this model is fine-tuned according to the target dataset named HAM10000 having seven skin classes. The FC layer is removed in the fine-tuning process and a new FC layer is added with seven outputs. Later, the FC layer is connected with the Softmax layer and output layer and trained using TL. The following parameters are initialized in the training process: the learning rate is 0.0001, epochs are 100, the minibatch size is 64, and the learning method is Stochastic Gradient Descent (SGD). Features are extracted from the average pooling layer, which is later utilized for the classification process. On this layer, the dimension of extracted features is *N* × 2048.

### 2.6. Feature Fusion

Feature fusion is an essential topic in pattern recognition, where multisource features are fused in one vector. The main purpose of feature fusion is to increase the object information for accurate classification. In this work, we consider the idea of a serial-based approach named modified serial-based feature fusion. The proposed fusion approach works in two sequential steps. In the first step, all features of vectors are fused in one matrix, and later on, a standard error mean- (SEM-) based threshold function is proposed.

Assume that *P* and *Q* are two function rooms on the sample size pattern Δ. The corresponding two characteristic vectors *δ* ∈ *P* and *γ* ∈ *Q* for an arbitrary sample are *ƒ* ∈ Δ. The serial-based feature combination of *ƒ* is defined as $\omega =\left(\begin{array}{c} \delta \\ \gamma \end{array}\right)$. Of course, if the vector feature *δ* is *n*-dimensional and *γ* is *m*-dimensional, then the combined serial feature *ω* is (*n*+*m*)-dimensions [45]. A serial combined feature space is created by combining all serially merged feature vectors of pattern samples of (*n*+*m*)-dimensions. The resultant *ω* vector has dimension *N* × 4096. After this step, SEM is computed of *ω* using the following formulation:

(11) $$\begin{array}{c} \text{SEM}=\frac{s}{\sqrt{n}},\\ s=\sqrt{\sum_{i=1}^{n}\frac{{\left(\omega_{i}-\text{Mean}\right)}^{2}}{n-1}},\\ \text{Thr}=\left\{\begin{array}{cc} \text{Fus}\left(i\right), & \text{for }\omega_{i}\geq \text{SEM,}\\ \text{Nfus}\left(j\right), & \text{elsewhere,} \end{array}\right. \end{array}$$

where Thr denotes the threshold function, Fus(*i*) is fused feature vector of dimension *N* × 2506, Nfus(*j*) is a feature that is not considered in the fused vector, and *s* is a standard deviation value. The output of this step is further refined in the feature selection step, as given below.

### 2.7. Feature Selection

The goal of feature selection is to reduce input variables when a predictive model is developed. This process minimizes the computational time of a proposed system and improves classification accuracy. In this work, a new heuristic search-based feature selection method is proposed named skewness-controlled SVR. In the first step, a skewness feature vector is extracted from the fused vector Fus(*i*). This step aims to find the likelihood of the features falling in the specific probability distribution. Mathematically, skewness is computed as follows:

(12) $$\begin{array}{c} \text{Skew}=\frac{3\bar{\text{Fus}\left(i\right)}-\text{Median}}{s}, \end{array}$$

where Skew is the skewness feature vector, $\bar{\text{Fus}\left(i\right)}$ is the mean value of the fused feature vector, and *s* is the standard deviation. Using this skewness value, a threshold function is defined to select features at the first stage.

(13) $$\begin{array}{c} \text{Thr }1=\left\{\begin{array}{cc} \text{Sel}\left(i\right), & \text{for Fus}\left(i\right)\geq \text{Skew,}\\ \text{Ignore}, & \text{elsewhere}. \end{array}\right. \end{array}$$

Using this threshold function, features are selected at the initial phase. The selected features of this phase are later validated using a fitness function Support Vector Regression (SVR). The SVR is formulated as follows.

Assume that the dataset for training *Q* comprises the instances *q*, each having an attribute *u*_*i*_, an associated class, and *v*_*i*_. *u*_*i*_ ∈ Sel(*i*) is a selected feature and *v*_*i*_ represents labels; i.e., {(*u*_1_, *v*_1_),  (*u*_2_, *v*_2_),…, (*u*_*q*_, *v*_*q*_)}. On the dataset *D*, *b* is a bias, and the linear function *f*(*x*) may be defined as follows:

(14) $$\begin{array}{c} f\left(u\right)=\delta_{1}u_{1}+\;\delta_{2}u_{2}+\cdots +\delta_{d}u_{d}+b, \end{array}$$

where the weight *δ*_*i*_ is defined as input space *S*^*d*^; i.e., *δ*_*i*_ ∈  *S*^*d*^. The maximum margin size is determined by the Euclidean weight (‖*Y*‖). The flatness, therefore, requires a minimum weight standard in the case of the following equation. Here, the definition of (‖*Y*‖) is

(15) $$\begin{array}{c} {\left\|Y\right\|}^{2}=Y_{1}^{2}+Y_{2}^{2}+\cdots +Y_{d}^{2}. \end{array}$$

Each training data error may be represented as 〈*u*_*i*_, *v*_*i*_〉.

(16) $$\begin{array}{c} {\text{Err}}_{i}\left(u_{i}\right)=v_{i}-\left(\delta_{i}u_{i}+b\right). \end{array}$$

If there is error Err_*i*_(*u*_*i*_), the deviation is permitted to be within it, and the previous equation may be expressed as *ŋ*.

(17) $$\begin{array}{c} v_{i}-\left(\delta_{i}u_{i}+b\right)\leq ŋ,\\ \left(\delta_{i}u_{i}+b\right)-v_{i}\leq ŋ. \end{array}$$

Using these two equations, the minimization issue for *δ* can be formulated as follows:

(18) $$\begin{array}{c} \text{minimized}:\frac{1}{2}{\left\|Y\right\|}^{2}, \end{array}$$

subject to

(19) $$\begin{array}{c} v_{i}-\left(\delta_{i}u_{i}+b\right)\leq ŋ,\\ \left(\delta_{i}u_{i}+b\right)-v_{i}\leq ŋ. \end{array}$$

The restrictions of the above equation imply that the function *f* corresponds to all pairings (*u*_*i*_, *v*_*i*_) with a deviation of *ŋ*. However, the assumption is not accepted in all instances when the slack variables *𝔷*_*i*_*𝔷*_*i*_^*∗*^ are neither required nor necessary in case of violation of the assumption. The optimization problem may be reformulated using slack variables as follows:

(20) $$\begin{array}{c} \text{minimize}:\;\frac{1}{2}{\left\|Y\right\|}^{2}+C\sum_{i=0}^{d}\left(z_{i}+z_{i}^{*}\right), \end{array}$$

subject to

(21) $$\begin{array}{c} \forall_{i}=v_{i}-\left(\delta_{i}u_{i}+b\right)\leq ŋ+z,\\ \forall_{i}=\left(\delta_{i}u_{i}+b\right)-v_{i}\leq ŋ+z^{*},\\ \forall_{i}:z_{i}\geq 0,\\ \forall_{i}:z_{i}^{*}\leq 0, \end{array}$$

where *C* is the penalty constant, which does not meet the constraints. It also helps in reducing overfitting. The Kernel is defined by the input data *K*(*u*_*i*_, *u*_*j*_) and can substitute the occurrence of the dot product between the tuples to avoid the dot product on a data tuple changed. All computations are therefore done in the original input areas. In this work, a radial basis Kernel/Gaussian function is utilized:

(22) $$\begin{array}{c} K\left(u_{i},u_{j}\right)=\exp-\frac{\left({\left\|u_{i},u_{j}+1\right\|}^{2}\right)}{2\rho^{2}}. \end{array}$$

The accuracy is computed using SVR, and if accuracy is less than the target accuracy value, then Sel(*i*) is again updated. This process is continued until the maximum number of iterations is performed. In this work, the target accuracy is 90%, and the numbers of iterations are 5. Following this process, a feature vector is obtained called the best-selected feature vector of dimension *N* × 1456 and further fed to supervised learning algorithms for final classification.

## 3. Experimental Results and Discussion

The proposed method is evaluated on the augmented HAM10000 dataset. Dataset is divided into 70 : 30, where the 70% data is used for the training of a model, and the rest of the 30% is utilized for the testing process. The other training hyperparameters; for example, epochs are 100, the minibatch size is 64, and the learning rate is 0.0001. The 10-fold method was carried out for cross-validation [46]. Seven performance measures are used for the experimental process: recall rate, precision rate, false-negative rate (FNR), Area under Curve (AUC), accuracy, time, and *F*1-score. The proposed method is implemented in MATLAB 2020b, Corei7, with a RAM 16GB and 8GB graphics card.

### 3.1. Results

In this section, the proposed method results are described in numerical values (Tables) and confusion matrixes. Total ten classifiers are utilized for the experimental process, such as Linear Support Vector Machine (LSVM), Quadratic SVM (QSVM), Cubic SVM (CSVM), Medium Gaussian SVM (MGSVM), Cosine *K*-Nearest Neighbor (CKNN), Weighted KNN (WKNN), Coarse KNN (CKNN), Ensemble Subspace Discriminative (ESD), Ensemble Boosted Tree (EBT), and Ensemble Subspace KNN (ESKNN). Five experiments are performed for the validation of the proposed framework such as (i) Experiment # 1: classification using fine-tuned ResNet-50 CNN model, (ii) Experiment # 2: classification using Fine-Tuned ResNet-101CNN model, (iii) Experiment # 3: perform features fusion of Fine-Tuned ResNet-50 and ResNet-101 CNN models, and (iv) Best Features (BF) selection.

#### 3.1.1. Experiment # 1

In the first experiment, features are extracted using fine-tuned ResNet-50 CNN model, and results are computed. The augmented dataset was used for the experimental process. The results of this experiment are given in Table 1. CSVM has the highest accuracy of 92.7% in this table, with computational time 1190.3 (sec).  Figure 12 shows the confusion matrix of CSVM for this experiment. In this figure, the diagonal values represent the correct predicted values such as AKIEC (96%), BCC (93%), BKL (87%), DF (97%), MEL (86%), NV (94%), and VASC (99%), respectively. Moreover, the recall rate is 93.14, the precision rate is 93.14, and F1-score is 93.14%, respectively. Compared with the rest of the classifiers, it is noticed that the CSVM showed better classification accuracy. Moreover, the computational time of each classifier is also noted and plotted in Figure 13. This figure shows that the CKNN has the lowest computational time of 274.55 (sec).

#### 3.1.2. Experiment # 2

Table 2 presents the results of fine-tuned ResNet-101 CNN features using the augmented HAM10000 dataset. This table shows that the best accuracy achieved by CSVM is 92.1%, with a computational time of 11321.1 (sec), recall rate is 92.7, the precision rate is 92.42, and F1-score is 92.56%, respectively.  Figure 14 shows the confusion matrix of CSVM. In this figure, the diagonal values represent the correct predicted values such as AKIEC (96%), BCC (92%), BKL (85%), DF (98%), MEL (86%), NV (93%), and VASC (99%), respectively. As given in this table, a few other classifiers are also implemented and show that the CSVM gives better accuracy. Moreover, the computational time is computed for each classifier, and the minimum noted time is 260.5 (sec) for the W-KNN classifier. The noted time is also plotted in Figure 15.

#### 3.1.3. Experiment # 3

In the next experiment, features are fused using the serial-based extended (SbE) approach. Results are given in Table 3. This table represents the best accuracy achieved by the ESD classifier of 95%, further demonstrating in a confusion matrix, given in Figure 16. This figure represents the correct predicted values such as AKIEC (97%), BCC (94%), BKL (89%), DF (98%), MEL (89%), NV (99%), and VASC (99%), respectively. The other computed measures are recall rate, precision rate, FNR, AUC, and F1-score of 95.0, 95.0, 5.00, 0.99, and 95.0%, respectively. The CSVM achieved the second-best accuracy of 94.9%, whereas the recall rate and precision rates are 95.0%. Comparison with the rest of the classifiers shows the superiority of the ESD classifier. Moreover, the computational time is also noted, as illustrated in Figure 17.

Compared with the results of this experiment with Tables 1 and 2, it is noticed that the fusion using the SbE approach significantly improves the classification accuracy. The limitation of this step increases computational time, which needs to be minimized.

#### 3.1.4. Experiment # 4

Finally, the proposed feature selection algorithm is applied on the fused feature vector and achieved an accuracy of 91.7% on the ESD classifier, where the computational time is 1367 (sec), given in Table 4. The recent time was 4118 (sec), which is significantly minimized after the selection algorithm. This table also showed that the proposed accuracy decreases, but on the other side, it helps to minimize the computational time. The accuracy of the ESD classifier is further verified using a confusion matrix given in Figure 18. In this figure, the diagonal values represent the correct predicted values such as AKIEC (94%), BCC (91%), BKL (85%), DF (93%), MEL (83%), NV (97%), and VASC (99%), respectively.

The F1-score-based analysis is also conducted and plotted in Figure 19. In this figure, it is illustrated that the value of the F1-score is improved after the feature fusion process except the CKNN and EBT classifier. Moreover, the feature selection approach reduced the computational time but accuracy is degraded. Overall, the proposed framework performed well on the selected dataset. In the last, the proposed method accuracy is compared with some recent techniques, as given in Table 5. In this table, Khan et al. [7] presented a deep learning method for skin lesion classification. They used the HAM10000 dataset and achieved an accuracy of 88.5%. The recent best-reported accuracy was 91.5%, achieved by Sevli [47]. The proposed accuracy is 91.7% and 95% for the best feature selection approach and fusion approach. Based on this accuracy, it is noted that the proposed method showed improved accuracy.

## 4. Conclusion

In this work, a new framework is presented for multiclass skin lesion classification using deep learning. The proposed method consisted of a series of steplike data augmentation, feature extraction using deep learning models, the fusion of features, selection of parts, and classification. The experiment was performed on an augmented HAM10000 dataset. The number of experiments was performed, such as nonaugmented and augmented datasets, and achieved accuracy with a nonaugmented dataset of 64.36% using ResNet-50 and 49.98% using ResNet-101. The augmented dataset achieved an accuracy of 95.0% for feature fusion and 91.7% for feature selection. The results show that the augmentation process helps improve the classification accuracy for a complex dataset.

Moreover, the fusion process increases the performance but also increases the computational time. This process can be further refined through a feature selection process. However, according to the results, the feature selection process decreases the computational time and reduces accuracy. But from the overall comparison with recent techniques, feature fusion and feature selection technique both perform better than previous techniques. The new datasets ISBI 2020 and ISIC 2020 can be used for the experimental process in future work. Latest deep learning models can be used as feature extraction. Fusion can be performed using parallel approaches. The selection process can be refined, which not only reduces the time but also increases accuracy.

## Figures and Tables

**Figure 1:** Graph of infected and death cases of skin lesion.

**Figure 2:** Architecture of proposed methodology.

**Figure 3:** Sample skin lesion images of the HAM10000 dataset [7].

**Figure 4:** Flip operations in data augmentation.

**Figure 5:** A general structure of a CNN model for skin lesion classification.

**Figure 6:** Transfer learning-based training a new target model for the classification of skin lesions.

**Figure 7:** Residual identity mapping.

**Figure 8:** Architecture of ResNet-50.

**Figure 9:** Block diagram of fine-tuned ResNet-50.

**Figure 10:** Fine-tuned architecture of ResNet-101.

**Figure 11:** Transfer learning architecture with modified ResNet-101 model (*n* = 23 for ResNet-101; stride*∗S* and padding*∗P*).

**Figure 12:** Confusion matrix of CSVM using ResNet-50 model for HAM10000 dataset.

**Figure 13:** Time plot for fine-tuned ResNet-50 CNN model using augmented HAM10000 dataset.

**Figure 14:** Confusion matrix of CSVM using ResNet-101 model for HAM10000 dataset.

**Figure 15:** Time plot for fine-tuned ResNet-101 CNN model using augmented HAM10000 dataset.

**Figure 16:** Confusion matrix of ESD using ResNet-50 and ResNet-101 model for HAM10000 dataset.

**Figure 17:** Time plot for the fusion of ResNet-50 and ResNet-101 using augmented dataset (HAM10000).

**Figure 18:** Confusion matrix of ESD classifier using a proposed feature selection algorithm.

**Figure 19:** F1-score-based analysis of middle steps like ResNet-50, ResNet-101, and fusion.

**Table 1:** Classification accuracy of fine-tuned ResNet-50 deep features using augmented HAM10000 dataset.

Classifier	Recall rate (%)	Precision rate (%)	FNR (%)	AUC	Accuracy (%)	Time (sec)	*F*1-score (%)
LSVM	86.42	86.85	13.57	0.988	86.5	742.5	86.63
QSVM	92.00	92.14	8.00	0.992	91.7	1046.1	92.07
**CSVM**	**93.14**	**93.14**	**6.858**	**0.994**	**92.7**	1190.3	**93.14**
MGSVM	89.57	90.00	10.42	0.988	89.3	1906.8	89.78
CKNN	53.25	65.28	46.75	0.898	60.8	**274.5**	58.65
CKNN	80.42	79.00	19.57	0.967	78.7	287.6	79.70
WKNN	85.14	84.42	14.85	0.98	83.6	262.3	84.78
ESKNN	93.14	92.57	6.858	0.99	92.3	4514.7	92.85
EBT	55.28	86.71	44.71	0.974	57.1	1546.0	86.49
ESD	86.28	57.00	13.71	0.85	86.1	839.8	56.12

The bold value represents best ones.

**Table 2:** Classification accuracy of fine-tuned ResNet-101 deep features using augmented HAM10000 dataset.

Classifier	Recall rate (%)	Precision rate (%)	FNR (%)	AUC	Accuracy (%)	Time (sec)	*F*1-score (%)
LSVM	86.00	86.28	14.00	0.98	85.5	746.2	86.14
QSVM	91.57	91.71	8.428	0.992	91.1	1010.2	91.64
**CSVM**	**92.71**	**92.42**	**7.285**	**0.992**	**92.1**	11321.1	**92.56**
MGSVM	89.42	89.42	10.57	0.988	88.9	1919.4	89.42
CKNN	78.87	77.85	21.14	0.961	77.2	268.2	78.36
CKNN	58.42	63.00	41.27	0.887	58.9	263.6	60.62
WKNN	84.85	84.00	15.14	0.977	83.3	**260.5**	84.42
EBT	56.57	56.57	43.42	0.855	57.2	1544.5	56.57
ESKNN	80.28	92.28	19.71	0.99	92.1	4590.9	85.86
ESD	85.85	86.28	14.14	0.98	85.6	821.79	86.06

The bold value represents best ones.

**Table 3:** Classification results using SbE approach-based deep features fusion on augmented HAM10000 dataset.

Classifier	Recall rate (%)	Precision rate (%)	FNR (%)	AUC	Accuracy (%)	Time (sec)	*F*1-score (%)
LSVM	92.71	92.85	7.285	0.992	92.50	1303.8	92.78
QSVM	94.85	94.85	5.142	0.997	94.80	2400.4	94.75
CSVM	95.00	95.00	5.00	0.854	94.90	2868.5	95.00
MGSVM	92.85	93.14	7.142	0.995	92.60	4501.6	92.99
CKNN	61.71	73.14	38.28	0.910	62.20	562.0	66.94
CKNN	84.14	83.57	15.85	0.975	82.60	550.5	83.85
WKNN	83.42	84.57	16.27	0.971	82.10	**530.7**	83.99
**ESD**	**95.00**	**95.00**	**5.00**	**0.997**	**95.00**	**4118.2**	**95.00**
FKNN	88.14	87.57	11.85	0.931	87.00	543.2	87.85
EBT	62.00	62.22	38.00	0.855	62.80	69886.0	62.11

The bold value represents best ones.

**Table 4:** Classification results using proposed feature selection algorithm on augmented HAM10000 dataset.

Classifier (ESD)	Recall rate (%)	Precision rate (%)	FNR (%)	AUC	Accuracy (%)	Time (sec)	*F*1-score (%)
500	78.42	79.28	21.57	0.954	78.3	102.4	78.85
1000	64.85	66.71	35.14	0.902	65.1	**132.5**	65.77
1500	87.14	87.57	12.85	0.978	86.8	406.0	87.35
2000	83.57	84.42	16.42	0.97	83.3	748.4	83.99
2500	89.71	90.14	10.28	0.984	89.5	1293.5	89.92
**3000**	**91.85**	**92.00**	**8.142**	**0.99**	**91.7**	**1367.6**	**91.92**

The bold value represents best ones.

**Table 5:** Comparison with existing techniques.

Reference	Year	Dataset	Accuracy (%)
[7]	2020	HAM10000	88.5
[48]	2020	HAM10000	86.1
[49]	2020	HAM10000	83.1
[30]	2021	HAM10000	85.50
[47]	2020	HAM10000	91.5
**Proposed (fusion)**	**2021**	**HAM10000**	**95.0**
**Proposed (feature selection)**	**2021**	**HAM10000**	**91.7**

The bold value represents best ones.

## Data Availability

The HAM10000 dataset is utilized in this work for the experimental process. The dataset is publically available at https://dataverse.harvard.edu/dataset.xhtml?persistentId=doi:10.7910/DVN/DBW86T.
